# Handwashing Practice among Elementary Schoolchildren in Urban Setting, Mongolia: A School-Based Cross-Sectional Survey

**DOI:** 10.1155/2022/3103241

**Published:** 2022-09-16

**Authors:** Munguntuul Enkhbat, Ganchimeg Togoobaatar, Oyunchimeg Erdenee, Asako Takekuma Katsumata

**Affiliations:** ^1^Graduate School of Comprehensive Human Sciences, University of Tsukuba, 1-1-1, Tennodai, Tsukuba, Ibaraki 305-8577, Japan; ^2^Department of Public Health Nursing, School of Nursing, Mongolian National University of Medical Sciences, Bayangol District, Ard Ayush Street, Ulaanbaatar 16081, Mongolia; ^3^Department of Global Health Nursing, Faculty of Medicine, University of Tsukuba, 1-1-1, Tennodai, Tsukuba, Ibaraki 305-8577, Japan; ^4^Tuberculosis Surveillance and Research Department, National Center for Communicable Diseases, NCCD Campus, Nam-Yan-Ju Street, Ulaanbaatar-13335, Mongolia

## Abstract

**Objectives:**

Handwashing with soap is the simplest, most affordable, and cost-effective preventative intervention for reducing the burden of communicable diseases, including the COVID-19. This study was aimed at investigating elementary schoolchildren's handwashing practice at two critical moments, namely, before eating and after using the toilet and its associated factors.

**Methods:**

The cross-sectional study was conducted at ten public secondary schools in Ulaanbaatar, Mongolia, between February and March 2019. Data were collected from all fifth-grade children's parents at the selected schools by using a self-reported questionnaire. Descriptive and multiple regression analyses were conducted using STATA/MP version 13.0.

**Results:**

A total of 1507 parents/guardians of 5^th^-grade school children participated. Reported schoolchildren's handwashing practice for both critical moments was 50.1%. It was significantly associated with female gender (adjusted odds ratio [AOR] = 0.56 (95%CI = 0.45, 0.70)), number of siblings (AOR = 0.72 (95%CI = 0.61, 0.80)), and availability of handwashing amenity at school (AOR = 1.1595%CI = 0.86, 1.42)). Only 34% of children wash their hands with soap at school, and the most common reasons for skipping handwashing were an absence of soap (23.9%), lack of sink (14.5%), and the use of hand sanitizer (19.7%).

**Conclusions:**

The school children's handwashing practice at two critical moments is considerably low. The main disabling factors of regular handwashing at school included insufficient handwashing facility and soap. Therefore, promoting HW facilities and innovative and participatory education for elementary schoolchildren should be prioritized.

## 1. Introduction

Despite global efforts, infectious diseases, particularly pneumonia and diarrhea, continue to be the leading cause of mortality and morbidity among children in low- and middle-income countries [1]. Handwashing (HW) with soap is the simplest, most affordable, and cost-effective preventative intervention for reducing the burden of these diseases [2]. It has been recommended as a critical prevention measure against the novel coronavirus disease (COVID-19) [3, 4]. Systematic reviews of the health effects of HW with soap reported an estimated 23% to 48% and 21% of risk reduction in diarrhea [5] and acute respiratory infections [6], respectively. HW among schoolchildren also has a significant social and economic impact on the family and society by reducing school absenteeism and the loss of caregivers' workdays [7–10].

Although there are health and social benefits, HW practice remains significantly low globally. HW during two critical moments, namely, before eating and after toilet use, is the most used indicators of the practice in the population [11]. Studies among school children in low- and middle-income countries reported that 7% to 15% wash their hands after toilet use. Poor HW practices were associated with inadequate facilities in terms of both quantity and quality, lack of water supply and soap, and absence of norms or culture at the school or in the community [12]. Globally, approximately half of the schools do not have HW facilities with water and soap [11].

Mongolia is a lower-middle-income country where respiratory infection and diarrhea have steadily remained the leading causes of child morbidity and mortality [13]. Sanitation and hygiene are crucial public health challenges as 60% of households live in underdeveloped infrastructural and poor hygiene environments, including outdoor latrines and noncentralized water supply sources [8]. According to the WHO/UNICEF Joint Monitoring Program for Water Supply, Sanitation, and Hygiene (WASH), the national coverage [14] of basic hygiene services defined as HW facilities with water and soap in Mongolian schools was 41.4% in 2016. Moreover, 8 to 11% of high schoolchildren never or rarely wash their hands before eating and after using the toilet [15]. HW practice data among elementary school children in Mongolia is scarce. As they receive formal HW education at school, it is crucial to explore the practice among this population. Furthermore, acquiring proper HW practice at a young age is essential, as they are likely to be carried into adulthood [16, 17].

Therefore, this study was aimed at exploring elementary schoolchildren's HW practice and the associated factors and constraints.

## 2. Methods

### 2.1. Study Setting

This school-based cross-sectional study was conducted in Ulaanbaatar, the capital of Mongolia. The city is divided into nine districts with similar residential characteristics, namely, “*apartment/urban*” and *“ger/suburban*”(traditional dwellings). More than half of the 3,238,500 inhabitants of the country reside in Ulaanbaatar [18, 19]. The prevalence of infectious diseases in the city is higher than the national average, which may be attributed to high population density, unsanitary conditions, and unhygienic practices, specifically in the ger areas [19, 20].

In Mongolia, 12-year secondary education is provided primarily through public schools. In most cases, elementary (grades 1-5), lower (grades 6-9), and upper (grades 10-12) secondary education levels are combined into one school, with an average of 1,500 to 2,000 children. The Ministry of Education and Science is the central administrative body that formulates the national education policy and sets the standards and curriculum. Therefore, the budget finance and infrastructure of the schools are similar, specifically in the capital city [21].

This study was conducted in one of the six central districts of Ulaanbaatar, which accounted for 16% (22/134) of public schools in the city [22]. The district population in 2018 was 145,335, approximately 10% of the Ulaanbaatar population.

### 2.2. Study Participants

This study is a part of a cluster-randomized trial on the effectiveness of exercise interventions for children's academic achievement and health. Study sampling and methodology details of the original study have been written elsewhere [23, 24]. Briefly, ten public schools were recruited from 22 schools in the selected district. Schools that provided only upper secondary education (*n* = 10) or those for children with special needs (*n* = 2) were excluded. All fifth-grade children at the recruited schools were eligible. After identifying the children, the researchers sent an invitation letter with informed consent for their parents. In our study, the participants were parents or primary guardians who provided written informed consent.

### 2.3. Data Collection

Data were collected between February and March 2019 using a self-reported questionnaire. The questionnaire comprised three sections and 23 questions: (a) sociodemographic characteristics including parents' education, number of family members, household income, housing condition, and the child's age and sex; (b) children's HW practice and frequency, HW at two critical moments, and presence of infectious illness two weeks prior to the study; and (c) HW facilities at school, reasons to skip regular HW, and provision of HW education.

This study used sociodemographic questions from the National Household Survey of Mongolia [22]. The most commonly used school survey questionnaire developed by the UNICEF/WHO to explore children's HW practice in Mongolia and other countries was adapted [25–27]. The forward and back translations were conducted by independent translators fluent in English and Mongolian. The chief investigator and two researchers synthesized and revised the translated versions. Content and face validity of the questionnaire were conducted by involving schoolteachers and a small group of schoolchildren.

Data were collected by ten senior university students who attended a five-day training workshop of the main study that covered the aim of the study, research ethics, content of questionnaires, interview instructions, and guides developed by the research team. The questionnaire was sent to the primary guardians or parents in an enclosed envelope. They were asked to return it after completion.

### 2.4. Data Analysis

Children's HW practice was the independent variable of this study. It was defined based on the response to HW before eating and after using the toilet. On a 4-point Likert scale ranging from “always” to “never,” the children were asked to respond whether they washed their hands before and after. The responses “always” or “usually” for both moments were categorized as “washers,” and other responses as “nonwashers.”

The explanatory variables were sex, number of children in the family (≤2 or ≥3 children), housing type (ger/simple house or apartment), monthly household income (below; above 700,000 MNT was equal to about USD 280), maternal education (≤10; ≥11 years), HW education at school (no/yes), school area (urban/apartment vs. suburban (ger and mixed area)), and availability of HW amenities and sink (not available/only sink or soap available/both available).

Descriptions of the sociodemographic characteristics, HW practices, and barriers at school were presented as percentages, frequency (*n*), or mean (standard deviation, SD) values. Univariate and multivariable logistic regression analyses were performed to identify factors associated with HW practice and expressed as odds ratios (ORs) and adjusted odds ratios (AORs) and their corresponding 95% confidence intervals (CIs). The statistical significance threshold was set at *p* < 0.05. Data analysis was performed using STATA/MP version 13.0 (STATA Corp. LP, College Station, TX, USA).

### 2.5. Ethical Consideration

This study was approved by the ethics committee of the Mongolian National University of Medical Sciences (approval no. 3/18/2018-12-21). Written informed consent was obtained from the parents or primary guardians of the children.

## 3. Results

There were 55 fifth-grade classes in the 10 participating secondary schools. On average, there were six (range: 4 to 8) fifth-grade classes and 150 ± 23.6 (93-231) schoolchildren per school. The number of children per class was 27 ± 8.5 (28-71). The questionnaire was distributed to 1,836 children, and 1,693 were returned. A total of 1,507 completed questionnaires were analyzed.

### 3.1. Characteristics of Participants

Sociodemographic and school characteristics are shown in Table 1. The mean age of the schoolchildren was ten (±0.32) years. Half of them were boys and had more than two siblings. Over 60% attended schools in urban areas.

Approximately 55% of the mothers had more than ten years of education, 54.8% of households lived in apartments, and 63.1% reported more than 700,000 MNT as household income.

### 3.2. Children's HW Practice

As shown in Table 2, school children's HW practice was assessed by two critical moments. Among 1458 children, 25.7% and 35.3% reported that they wash their hands “always” and “usually” before eating, whereas 22.8% and 47.8% of 1,439 children washed their hands “always” and “usually” after the toilet, respectively.

After excluding missing data on HW practice questions, the data of 1,374 children remained for further analysis. Half (*n* = 690) of those reported that they wash their hands “always” or “usually” before and after and were categorized as “washers.” About 20% reported they wash their hands “sometimes” or “never,” whereas 30.2% reported “always” or “usually” for one of the moments. These two groups are referred to as “nonwashers” as shown in Figure 1.

### 3.3. Associated Factors with Schoolchildren's HW Practice

The analysis of school children's HW practice and associated factors is shown in Table 3. Boys and children who have more than three siblings were less likely to wash their hands frequently at the two critical moments compared to girls (adjusted odds ratio [AOR] = 0.56 [95% confidence interval [CI] = 0.45, 0.70]) and those with fewer siblings (AOR = 0.76 [95%CI = 0.61, 0.94]), respectively. Children's HW practice at these two critical moments were significantly associated with the availability of sink and soap at school (AOR = 1.42 [95%CI = 1.04, 1.88]). There was no significant association between HW practice and housing type, income, HW education at school, or school location. One-third of 1,507 (33.5%) children fell sick two weeks before the study, and the majority (81%) indicated respiratory symptoms. However, no significant association was found between illness and HW practice in our study (data not shown).

### 3.4. HW Practice at School and Reasons for Skipping

Schoolchildren's HW practice at school was assessed by the frequency, soap usage, HW facility location, and barriers of regular HW (Table 4). The reported frequency of fewer than six times per day among 1,507 children was 84.9%. A total of 1,492 participants completed the question “Did your child wash their hands today at school?” and among them, 34.1% washed their hands with soap, whereas 13.0% did not wash their hands at all. Approximately 85% of 1,507 children reported that they washed their hands in the toilet. HW was skipped at school because of the absence of soap (23.9%), lack of sink (14.5%), and use of hand sanitizer (19.7%). About 12% of 1,485 respondents specified other reasons for skipping HW such as broken, dirty sinks or bad-tempered school workers (data not shown).

Most children (75.2%) attended HW education classes, and 56.1% reported a lack of HW amenities at schools.

## 4. Discussion

To the best of our knowledge, this is the first study with a considerably large sample of elementary school children focused on HW practice and their associated factors in an urban setting in Mongolia. HW practice is a significant school health and infection prevention concern, as the school environment has intense person-to-person contact levels that are susceptible to infection and spread to the community. The study findings are crucial to promoting frequent and proper HW practice among schoolchildren during the two critical moments, specifically during COVID-19 [5, 6, 28–35].

This study recruited 1,507 fifth-grade schoolchildren who attended public schools (*n* = 10) in one of the nine districts of Ulaanbaatar. Among the 1,374 children who completed the questionnaire, 19.7% and 30.2% reported that they washed their hands “sometimes” or “never,” respectively, for both or one of the two critical moments. Thus, approximately 50% of elementary school children were nonwashers or had poor HW practices. These findings are similar to those of a previous WHO school-based survey in Mongolia conducted at 59 public schools in 2013. A total of 5,393 children aged 12 to 18 years participated in the study, and 25.2% and 26.9% had “never” and “sometimes” washed their hands, respectively, before eating and after toilet use [15]. Our study findings indicated poor HW practices among Mongolian elementary schoolchildren. The possible explanations could be the low priority and intensity of HW education, the traditional teaching approach, lack of hygiene facilities, poor communication between school and community, and lack of parental guidance. These factors have been documented in previous studies conducted in similar countries [12, 36].

This study was aimed at identifying the factors related to HW practice among elementary school children, such as sex, number of children in the family, housing type, monthly household income, school location, and availability of HW education and amenities at school. The results of this study indicated that boys were less likely to wash their hands than girls (AOR = 0.59 [95% CI 0.45, 0.70]). A similar finding of sex differences in HW practice has been reported in school-based studies conducted in Zambia and Mexico [37, 38]. A school-based randomized controlled trial study in Zambia examined the effectiveness of a soap-on-a-rope intervention on HW practice with soap by recruiting 50 schools and 10,732 children and found boys were less likely to wash their hands in both control and intervention groups at baseline (AOR = 0.72 [95%CI = 0.66, 0.80]) [37]. Another study of school nurse inspections on the availability of supplies in Mexico found that girls' bathrooms had a significantly higher probability of being supplied with soap and hand dryers or towels [39].

In our study, children with more than two siblings were significantly less likely to wash their hands (AOR = 0.76 [95%CI = 0.61, 0.94]). A similar finding reported in the previous study in Korea suggested that when the number of children increases, parents' or guardians' guidance and time for the child's education and enforcing health behaviors will decrease [40].

In this study, 65.6% of 1,507 children reported that they wash their hands three to five times daily, and 15% washed their hands more than six times. This finding suggests that HW frequency among children was insufficient compared to the recommended frequency of ten times per day by the WHO/UNICEF Joint Monitoring WASH program [41]. This study also found that the availability of HW sinks, soaps, and insufficient time were the most common reasons for skipping HW at school. Only 32.9% of children reported that HW facilities with water and soap were available. The main HW place was the toilet. Only 9.2% of children washed their hands in the classroom, which implies that many children could not wash their hands before school lunch. Similar to the UNICEF analysis [42] of the situation of Mongolian children in 2014, our study suggested that insufficient facilities and lack of soap supply and time are key constraints to frequent and proper HW at school. During the last two decades, most schools in Ulaanbaatar have been overcrowded (38-54 children per class), with limited sanitation facilities [15]. The Mongolian National WASH guideline states that the sink-to-student ratio is 1 : 40, which corresponds to the minimum standard by the WHO [27]; however, 25% of public schools have not met the standards [43]. This indicates that the Mongolian government has to take action to improve sanitation infrastructure, construct new schools or expand school areas, and reinforce guidelines and policies.

In our study, 76.6% of children attended the HW education class; however, half of them reported insufficient HW practice. This may indicate the ineffectiveness of the promotion and provision of health education among children. In Mongolia, a 45-minute session on HW education by the national curriculum, which is primarily a knowledge-based and didactic teaching approach, is provided for fourth-grade children by the class teachers. Teachers' overload in teaching activities has been widely documented [44]. Shortage and limited availability of resources, including teaching aids [36, 45] and traditional teaching approaches, are ineffective in acquiring skills and changing behaviors [46]. Suggested effective educational interventions to improve schoolchildren's HW are child-centered, participatory, and practical learning education that involves innovative and low-cost applications with soap such as soap-on-a-rope [37], soap placed in the net hanging on the faucet, interactive, participatory HW education, user-friendly printed educational and HW guidelines [47–49], and school nurses' regular inspections for HW facilities and supplies [38]. Therefore, it is necessary to explore effective and feasible interventions to improve health practice and hygiene facilities in Mongolian schools.

Along with a large sample of elementary schoolchildren and a valid questionnaire, this study had a few limitations. First, as this was a cross-sectional study; causal relationships for all variables related to the study indicators could not be determined. Second, a self-reported questionnaire regarding HW practice was used. Proper HW practice is a socially desirable behavior; thus, self-response would be over-reported.

## 5. Conclusion

Our findings suggest that schoolchildren's HW practice at two critical moments are considerably low (50.1%). Male gender, number of household children, and availability of handwashing amenity at school were associated factors with poor handwashing practice. The main barriers to regular HW practice at school are insufficient facilities and soaps. Therefore, promoting HW facilities and interventions should be prioritized. Most (76.6%) children reported receiving formal HW education at school, but the application of the practice was low. Consequently, Mongolian education policymakers should consider innovative and participatory HW education for elementary schoolchildren.

## Figures and Tables

**Figure 1:** Children's handwashing practice for two critical moments (*N* = 1374). Note: washer is defined as one who washes hands always or usually both before eating and after using the toilet; nonwasher is defined as one who washes hands always or usually at only one of the critical moments or is not a regular washer at both moments.

**Table 1:** Characteristics of the study participants.

Characteristics	*n*	%
Children's sex (*n* = 1507)		
Girls	752	49.9
Boys	755	50.1
Children's age [mean (SD)]	1502	10 (0.3)
Numbers of children in the family (*n* = 1500)		
≤2 children	774	51.6
≥3 children	726	48.4
Maternal education (*n* = 1328)		
≤10 years	505	38.0
≥11 years	823	54.6
Housing type (*n* = 1501)		
Apartment	826	55.0
Ger/simple house	675	45.0
Household monthly income (*n* = 1490)		
≤700,000 MNT	539	36.1
≥700,001 MNT	951	63.8
School residential area (*n* = 1507)		
Apartment/urban area	896	59.5
Ger/suburb area	611	40.5
Handwashing educational class (*n* = 1447)		
Yes	1089	75.2
No	358	24.7
Availability of handwashing amenity at school (*n* = 1439)		
Sink and soap both available	474	32.9
Only sink or soap available	157	10.9
Not available	808	56.1

MNT: Mongolian Tugrik. 700,000 MNT was equivalated to 280 USD.

**Table 2:** Children's handwashing frequency at two critical moments.

	*n*	%
Handwashing before eating (*n* = 1458)		
Always	376	25.7
Usually	515	35.3
Sometimes	442	30.3
Never	125	8.5
Handwashing after toilet (*n* = 1439)		
Always	329	22.8
Usually	688	47.8
Sometimes	295	20.5
Never	127	8.8

**Table 3:** Factors associated with handwashing practices among elementary school children (*N* = 1374).

Characteristics	Handwashing at the most critical moments						
	Washers (*n* = 684)		Non-washers (*n* = 690)		OR	AOR	(95% CI)
	*n*	%	*n*	%			
School children's sex							
Girls	390	56.5	290	42.4	1	1	
Boys	300	43.5	394	57.6	0.56^∗∗∗^	0.59	(0.45–0.70)^∗∗∗^
Numbers of children in the family							
≤2 children	381	55.2	334	48.8	1	1	
≥3 children	309	44.8	350	51.0	0.76^∗^	0.76	(0.61–0.94)^∗^
Housing type							
Ger/simple house	297	43.1	302	44.1	1	1	
Apartment	393	56.9	382	55.8	1.03	1.13	(0.89–1.46)
Household monthly income							
≤700,000 MNT	441	63.9	446	65.2	1	1	
≥700,001 MNT	249	36.1	238	34.8	1.04	1.10	(0.85–1.42)
Handwashing education at school							
No	161	23.3	176	25.7	1	1	
Yes	529	76.6	508	74.2	1.11	1.10	(0.86–1.43)
Location of school							
Urban	432	32.6	412	60.2	1	1	
Suburban	258	37.4	272	39.8	0.85	0.85	(0.65–1.12)
School handwashing amenity							
Not available	243	35.2	276	40.3	1	1	
Sink or soap	266	38.5	264	38.6	1.15	1.11	(0.86–1.42)
Sink and soap both available	181	26.2	144	21.1	1.42^∗^	1.40	(1.04–1.88)^∗^

Note: ^∗∗∗^*p* < 0.001; ^∗∗^*p* < 0.01; ^∗^*p* < 0.05.

**Table 4:** Elementary school children's handwashing practice at school.

	*n*	%
Frequency of handwashing per day (*n* = 1507)		
≤2 times	291	19.3
3-5 times	988	65.6
≥6 times	228	15.1
Handwashing at school (*n* = 1492)		
Wash hands with soap	508	34.1
Wash hands water only	574	38.4
Clean hands with sanitizer	216	14.4
Did not wash	194	13.0
Handwashing place (*n* = 1507)		
Classroom	138	9.2
Toilet	1277	84.7
Other places	92	6.1
Reasons for skipping handwashing (*n* = 1485)		
Soap was not available	356	23.9
Not enough sink	216	14.5
Cleaned their hands with sanitizer	294	19.7
No time to wash hands	197	13.2
Forget to wash hands	191	12.8
Not necessary	43	2.8
Other	188	12.6

## Data Availability

The data used to support the findings of this study are available from the corresponding author upon request.

## References

[1] GBD 2019 Diseases and Injuries Collaborators (2020). Global burden of 369 diseases and injuries in 204 countries and territories, 1990-2019: a systematic analysis for the Global Burden of Disease Study 2019. *The Lancet*.

[2] Hadaway A. (2020). Handwashing: clean hands save lives. *Journal of Consumer Health on the Internet*.

[3] Mushi V., Shao M. (2020). Tailoring of the ongoing water, sanitation and hygiene interventions for prevention and control of COVID-19. *Tropical Medicine and Health*.

[4] World Health Organization (2020). COVID-19 pandemic heightens the importance of handwashing with soap. *World Health Organization-Africa*.

[5] Freeman M. C., Stocks M. E., Cumming O. (2014). Systematic review: hygiene and health: systematic review of handwashing practices worldwide and update of health effects. *Tropical Medicine and International Health*.

[6] Aiello A. E., Coulborn R. M., Perez V., Larson E. L. (2008). Effect of hand hygiene on infectious disease risk in the community setting: a meta-analysis. *American Journal of Public Health*.

[7] Azor-Martínez E., Gonzalez-Jimenez Y., Seijas-Vazquez M. L. (2014). The impact of common infections on school absenteeism during an academic year. *American Journal of Infection Control*.

[8] Bharat D., Briones H., Lahiri S. (2006). Mongolia-Manual on Promotion of Hygiene and Sanitation in Ger Areas.

[9] Nwajiuba C. A., Ogunji C. V., Uwakwe R. C., David E. I. (2019). Handwashing practices among children in public schools in Imo State, Nigeria. *Global Journal of Health Science*.

[10] Umwangange M. L. (2016). The effectiveness of handwashing health education session on raising school children’s knowledge and skills of proper handwashing technique. A pre test-post test design. *Texile International Journal of Public Health*.

[11] WHO & UNICEF (2016). Core questions and indicators for monitoring WASH in Schools in the Sustainable Development Goals. http://www.who.int/about/licensing/copyright_form/en/index.html%0Ahttp://www.who.int/about/licensing/copyright_form/en/.

[12] Xuan L. T. T., Hoat L. N. (2013). Handwashing among schoolchildren in an ethnically diverse population in northern rural Vietnam. *Global Health Action*.

[13] Tsedenbal N., Tsend-Ayush A., Badarch D., Jav S., Pagbajab N. (2018). Influenza B viruses circulated during last 5 years in Mongolia. *PLoS One*.

[14] UNICEF Mongolia (2016). *Water, Sanitation and Hygiene (WASH)*.

[15] World Health Organization (2013). *Global School-Based Student Health Survey 2013*.

[16] Cevizci S., Uludag A., Topaloglu N., Babaoglu U., Celik M., Bakar C. (2015). Developing students’ hand hygiene behaviors in a primary school from Turkey: a school-based health education study. *International Journal of Medical Science and Public Health*.

[17] Mohamed N. A., Mohd Rani M. D., Tengku Jamaluddin T. Z. M. (2020). Effect of hand hygiene intervention on the absenteeism of pre-school children in Klang Valley, Malaysia: a quasi-experimental study. *World Journal of Pediatrics*.

[18] Mongolian Statistical Information Service (2010). *Population Statistic, 2010*.

[19] Ebright J. R., Altantsetseg T., Oyungerel R. (2003). Emerging infectious diseases in Mongolia. *Emerging Infectious Diseases*.

[20] Center for Health Development (2019). *Health Indicator*.

[21] Ministry of Education Culture and Sciences, Oxford Policy Management, & UNICEF (2020). *Review of education management information system (EMIS) that track individual student data*.

[22] National Statistics Organization of Mongolia (2018). *Economic and social situation of Ulaanbaatar city*.

[23] Takehara K., Ganchimeg T., Kikuchi A. (2019). The effectiveness of exercise intervention for academic achievement, cognitive function, and physical health among children in Mongolia: a cluster RCT study protocol. *BMC Public Health*.

[24] Takehara K., Togoobaatar G., Kikuchi A. (2021). Exercise intervention for academic achievement among children: a randomized controlled trial. *Pediatrics*.

[25] Burns J., Maughan-Brown B., Mouzinho Â. (2018). Washing with hope: evidence of improved handwashing among children in South Africa from a pilot study of a novel soap technology. *BMC Public Health*.

[26] Ergin A., Bostanci M., Önal Ö., Bozkurt A. I., Ergin N. (2011). Evaluation of students’ social hand washing knowledge, practices, and skills in a university setting. *Central European Journal of Public Health*.

[27] UNICEF, ACF, & Ministry of Education Cultura and Science, Ministry of Health and Sport, Ministry of Finance (2015). *Recommendations for implementation of kindergartens, secondary schools, dormitory water, sanitation, hygiene norms and requirements*.

[28] Blencowe H., Cousens S., Mullany L. C. (2011). Clean birth and postnatal care practices to reduce neonatal deaths from sepsis and tetanus: a systematic review and Delphi estimation of mortality effect. *BMC Public Health*.

[29] Curtis V., Cairncross S. (2003). Effect of washing hands with soap on diarrhoea risk in the community: a systematic review. *In Lancet Infectious Diseases*.

[30] Ejemot-Nwadiaro R. I., Ehiri J. E., Arikpo D., Meremikwu M. M., Critchley J. A. (2008). Hand washing promotion for preventing diarrhoea. *Cochrane Database of Systematic Reviews*.

[31] Ejere H. O., Alhassan M. B., Rabiu M. (2015). Face washing promotion for preventing active trachoma. *Cochrane Database of Systematic Reviews*.

[32] Filteau S. (2009). The HIV-exposed, uninfected African child. *In Tropical Medicine and International Health*.

[33] Greenland K., Cairncross S., Cumming O., Curtis V. (2013). Editorial: can we afford to overlook hand hygiene again. *In Tropical Medicine and International Health*.

[34] Isaac R., Alex R. G., Knox T. A. (2008). Malabsorption in wasting HIV disease: diagnostic and management issues in resource-poor settings. *Tropical Doctor*.

[35] World Health Organization (2009). *WHO Guidelines on Hand Hygiene in Health Care. First Global Patient Safety Challenge Clean Care Is Safer Care. World Alliance for Patient Safety*.

[36] Graves J. M., Daniell W. E., Harris J. R., Obure A. F. X. O., Quick R. (2011). Enhancing a safe water intervention with student-created visual aids to promote handwashing behavior in Kenyan primary schools. *International Quarterly of Community Health Education*.

[37] Naluonde T., Wakefield C., Markle L. (2019). A disruptive cue improves handwashing in school children in Zambia. *Health Promotion International*.

[38] Ramos M. M., Schrader R., Trujillo R., Blea M., Greenberg C. (2011). School nurse inspections improve handwashing supplies. *Journal of School Health*.

[39] White S., Thorseth A. H., Dreibelbis R., Curtis V. (2020). The determinants of handwashing behaviour in domestic settings: an integrative systematic review. *International Journal of Hygiene and Environmental Health*.

[40] Song I. H., Kim S.-A., Park W.-S. (2013). Family factors associated with children’s handwashing hygiene behavior. *Journal of Child Health Care*.

[41] United Nations Children’s Fund (UNICEF) and World Health Organization (2018). *Drinking water, sanitation and hygiene in schools: global baseline report 2018*.

[42] UNICEF, & Government of Mongolia (2014). *Analysis of the Situation of Children in Mongolia*.

[43] UNICEF Mongolia, & Ministry of Education Culture Science and Sport, Swiss Agency for Development and Cooperation (2017). *The current situation of water, sanitation, and hygiene in schools, kindergartens, and dormitories*.

[44] Ministry of Education and Sciences (2019). *The current situation of water, sanitation, and hygiene in schools, kindergartens, and dormitorie*.

[45] Grover E., Hossain M. K., Uddin S., Venkatesh M., Ram P. K., Dreibelbis R. (2018). Comparing the behavioural impact of a nudge-based handwashing intervention to high-intensity hygiene education: a cluster-randomised trial in rural Bangladesh. *Tropical Medicine and International Health*.

[46] Le Thi Thanh X., Thilde R., Luu Ngoc H., Anders D., Flemming K. (2013). Teaching handwashing with soap for schoolchildren in a multi-ethnic population in northern rural Vietnam. *Global Health Action*.

[47] Chittleborough C. R., Nicholson A. L., Basker E., Bell S., Campbell R. (2012). Factors influencing hand washing behaviour in primary schools: process evaluation within a randomized controlled trial. *Health Education Research*.

[48] Early E., Cantwall E., English J., Larson E. (1998). Effect of several interventions on the frequency of handwashing among elementary public school children. *American Journal of Infection Control*.

[49] Snow M., White G. L., Kim H. S. (2008). Inexpensive and time-efficient hand hygiene interventions increase elementary school children’s hand hygiene rates. *The Journal of School Health*.

